This article has been retracted.

# Fut7 Promotes Adhesion and Invasion of Acute Lymphoblastic Leukemia Cells through the Integrin/Fak/Akt Pathway

**DOI:** 10.1155/2022/1864116

**Published:** 2022-06-25

**Authors:** Fei He, Lijun Yi, Changcheng Lai

**Affiliations:** Department of Hematology and Oncology, Jiangxi Province Children's Hospital, Nanchang, Jiangxi 330006, China

## Abstract

**Purpose:**

To investigate the role and mechanism of N-fucosyltransferase VII (FUT7) in acute lymphoblastic leukemia (ALL).

**Methods:**

Bone marrow tissues were collected from patients with ALL and children with immune thrombocytopenic purpura (control) hospitalized in our hospital during the same period. Then, the FUT7 expression in bone marrow tissues was detected by qRT-PCR and western blotting. Human ALL cell strain Jurkat was cultured, and after knockdown or overexpression of FUT7, cell proliferation, apoptosis, adhesion and invasion were examined by MTT assay, flow cytometry, fibronectin adhesion assay and transwell, respectively; the protein expression level of integrin *α*5, integrin *β*1, p-FAK, and p-AKT was tested by western blotting.

**Results:**

The FUT7 expression was up-regulated in bone marrow cells of ALL patients. After knockdown of FUT7, the proliferation, adhesion and migration ability of ALL cells were significantly reduced, and apoptosis was increased, while the overexpression of FUT7 obtained the opposite results. Moreover, the overexpression of FUT7 also promoted the protein expression of integrin *α*5, integrin *β*1, p-FAK, p-AKT.

**Conclusion:**

FUT7 can promote the adhesion and invasion of ALL cells by activating the integrin/FAK/AKT pathway.

## 1. Introduction

Acute lymphoblastic leukemia (ALL) is a common heterogeneous hematologic tumor in childhood. In the United States, it is reported that the incidence of ALL has reached 1.7 per 100,000 population annually and over half of the diagnosed patients are 20 years old and younger [1]. Besides, ALL is characterized by impaired differentiation and proliferation of immature lymphoid cells in the bone marrow, peripheral blood, and extramedullary sites [2]. Over the years, the discussion of molecular mechanism of pathogenesis has been the focus of research for ALL. And also, a lot of progress has been gradually acquired in cytogenetics, molecular biology, and immunological factors, providing some references for the clinical treatment of ALL. As the routine treatment of ALL, systemic chemotherapy has serious side effects [3]. Therefore, further exploration of the pathogenesis of ALL as well as affecting factors for the prognosis is needed to provide more options for ALL treatment in clinical practice. In recent years, molecular targeted drugs have become the most promising therapeutic method in cancer therapy and can achieve stronger anti-tumor cell efficacy compared with cytotoxic chemotherapeutic drugs. Targeted therapy is characterized by effects on abnormal molecular mechanisms or abnormal angiogenesis in malignant tumors, but mild damage to normal cells [4]. It is reported that chemotherapy in combination with tyrosine kinase inhibitors has showed a significant improvement in prognosis and survival in children with ALL [5]. Furthermore, JAK/STAT inhibitors are a new and potentially effective molecularly targeted agent for the treatment of ph-like B-cell ALL [5]. The above suggests that molecularly targeted agents also have a good efficacy in the treatment of ALL.

Current studies have demonstrated that glycans present on the cell surface and in the tumor microenvironment have an important impact on key events in cancer development, such as cell adhesion to each other, cell-matrix interaction, immune monitoring, and intracellular signal transduction [6–8]. Protein glycosylation is an important processing and modification mode of proteins. Specifically, according to different glycosylation connection sites, protein glycosylation is mainly divided into N-glycosylation and O-glycosylation. Fucosylation is a special form of glycosylation, and the known fucosylation modifications include H antigen of the ABO blood group system and Lewis blood group antigen [9]. Fucosylation, reported to be widespread in cancer cells [10], is not only a post-translational modification but also involved in selectin-mediated leukocyte extravasation or lymphocyte homing, pathogen-host interactions, and signal transduction [11]. In a variety of pathological conditions, fucosylation level presents an abnormal state, such as inflammation and tumors [12]. Fucosyltransferases (FUTs) can catalyze the synthesis of fucose at the end of glycan chains, and 13 kinds of FUTs have been found now. N-fucosyltransferases, as one of the FUTs, are divided into 1-2, 1–3, and 1–6 fucosyltransferases according to their different catalytic glycosidic bonds [13]. Relevant studies have manifested that fucosyltransferases engage in many physiological and pathological processes, such as embryo implantation, immune response, and tumor development and metastasis [14–17]. FUT7 belongs to 1–3 fucosyltransferases and acts on N-acetylglucosamine to specifically synthesize sLeX [18]. Wang et al. [19] found that sLeX was the most highly expressed Lewis antigen in primary liver carcinoma (PLC), particularly in cases of poor differentiation and metastasis. For one thing, FUT7 has been verified to be highly expressed in a variety of malignancies and is associated with poor prognosis in patients. For another, FUT7 has been indicated to promote epithelial-mesenchymal transition and immune infiltration in bladder urothelial carcinoma [20]. Mechanistic investigations revealed that FUT7 catalyzed the *α*1,3-fucosylation of the epidermal growth factor receptor (EGFR) in follicular thyroid carcinoma (FTC) to promote the malignant transformation [18]. It has also been found that FUT7 controls cell cycle progression through the PLC*γ*/extracellular signal-regulated kinase signaling pathway and plays an important role in human hepatoma cell proliferation [21]. In addition, the high FUT7 expression also presents a poor prognosis in acute myeloid leukemia [22]. However, the expression and role of FUT7 in ALL have not been reported in many studies. Therefore, this study made an in-depth exploration for the effect and mechanism of FUT7 on ALL cells based on clinical samples and in vitro experiments.

## 2. Materials and Methods

### 2.1. Clinical Samples

Bone marrow samples from 30 children with ALL were collected from the specimen bank of our hospital. The specimens met the following conditions: pediatric patients who were (≤16 years of age) newly diagnosed with ALL and did not receive treatment. The diagnosis and classification of ALL were conducted based on the “Specifications for the Diagnosis and Treatment of Children with Acute Lymphoblastic Leukemia (2018 Edition).” Another 10 bone marrow samples (control) were collected from children with immune thrombocytopenic purpura (ITP) admitted to the hospital during the same period. All patients signed informed consent, and this study was approved by the Ethics Committee of Jiangxi Province Children's Hospital (No: JXSETYY-YXKY--20200044).

### 2.2. Cell Culture

Human ALL cell line Jurkat cells were purchased from Shanghai Bogoo Biological Technology Co., Ltd. Then, the cells were cultured in RPMI-1640 medium containing 10% fetal bovine serum (FBS, Gibco, USA) in an optimal culture environment at 37°C with a saturated humidity of 5% CO_2_. And the cell culture medium was replaced after 2-3 days, and passage was performed according to 1 : 2.

### 2.3. Cell Transfection

FUT7 shRNA (si-FUT7) and its negative control (shNC, 100 nM), and pEGFP-N3-FUT7 (FUT7) and its negative control (NC, 100 nM) were provided by GenePharma Company (Shanghai, China). The above lentiviral plasmids were transfected according to Lipofectamine 2000 reagent (Invitrogen, Carlsbad, CA, USA) when the cell fusion reached 70–80% in a six-well plate. After 6 h, the transfection medium was changed to a fresh medium and another 48-h culture was conducted.

### 2.4. qRT-PCR

Total RNA from cells and tissue samples was extracted by the TRIzol reagent (Invitrogen, Carlsbad, CA, USA). Reverse transcription was performed using a reverse transcription kit (TaKaRa, Tokyo, Japan), and all procedures were conducted according to the instructions of the kit. The gene expression was determined through a LightCycler 480 (Roche, Indianapolis, IN, USA) fluorescence quantitative PCR instrument, and reaction conditions were carried out according to the operating instructions of the quantitative fluorescence PCR kit (SYBR Green Mix, Roche Diagnostics, Indianapolis, IN). Thermal cycling parameters are shown as follows: 95°C for 10 s, followed by a total of 45 cycles of 95°C for 5 s, 60°C for 10 s, and 72°C for 10 s; the final extension was at 72°C for 5 min. Three replicates per reaction were set up for quantitative PCR. GAPDH was adopted for internal control. The 2^−ΔΔCt^ method was utilized for data analysis. The primer sequences used in this study were shown in Table 1.

### 2.5. Western Blotting

After the cells were treated with RIPA lysate (Beyotime Biotechnology, Shanghai, China) for 30 min, the centrifugation was conducted at 12,000 rpm for 15 min at 4°C to collect the supernatant proteins. Then, after the protein concentration was measured with the BCA kit (Beyotime Biotechnology, China), the corresponding volume of protein was added into the loading buffer to mix well (Beyotime Biotechnology, China). Subsequently, the proteins were heated in a boiling water bath for 5 min to achieve denaturation. Furthermore, after electrophoretic separation, the proteins were transferred to PVDF membranes and blocked using 5% skimmed milk for 60 min. Primary antibodies GAPDH (5174S, 1 : 1000, Cell Signaling, Boston, USA), FUT7 (18197-1-AP, 1 : 500, Proteintech, Wuhan, China), integrin *α*5 (^#^ 98204S, 1 : 1000, Cell Signaling, Boston, USA), integrin *β*1 (^#^ 9699S, 1 : 1000, Cell Signaling, Boston, USA), p-FAK (^#^ 8556S, 1 : 1000, Cell Signaling, Boston, USA), and p-AKT (^#^ 4060S, 1 : 1000, Cell Signaling, Boston, USA) were added respectively for incubation overnight at 4°C on a shaker. The next day, the membranes were washed three times for 10 min per time with TBST. Then, the membranes were transferred into secondary antibody (horseradish peroxidase-labeled goat anti-rabbit IgG, 1 : 5000, Beijing Kangwei Century Biotechnology Co., Ltd., China, Beijing) for 1-h incubation at ambient temperature. After that, the membranes were washed three times with TBST (10 min per time). After the developer was dropped on the membranes, a chemiluminescence imaging system (Bio-rad) was utilized for detection.

### 2.6. MTT Assay

The transfected Jurkat cells with good growth status were made into cell suspensions using the culture medium, and then, cell suspensions containing 5 × 10^3^ cells were added to each well of a 96-well cell culture plate. Then, the plate was placed in an incubator for cell culture. Subsequently, after 48 h, 10 *μ*L MTT solution at the concentration of 5 mg/mL was added to each well. And after static culture in a cell incubator for 4 h, the culture medium was discarded, and 100 *μ*L DMSO solution was added to each culture well to dissolve the crystals. Then, the absorbance of the solution in each well at 490 nm was measured using a microplate reader.

### 2.7. Apoptosis Detection

The transfected cells were seeded in a six-well plate at 2 × 10^5^ cells/well, and then, the cells were collected and washed using prechilled PBS. Next, the cells were resuspended by adding 1 × buffer and then mixed with 5 *μ*L annexin V or PI in the dark. After that, the cells were incubated in the dark at room temperature for 15 min. Then, 1 × buffer was added to resuspend the cells, and the apoptosis was detected using a flow cytometer.

### 2.8. Fibronectin Adhesion Assay

Fibronectin at 5 *μ*g/mL was preplated in a 12-well plate. After 2 h at ambient temperature, the cells were seeded into wells plated with fibronectin at a density of 1 × 10^5^ cells/well for 1-h incubation at 37°C. Then, PBS was applied to remove cells that were not adhered. After fixation with 4% paraformaldehyde for 1 h, the cells were stained with 0.2% crystal violet for 1 h. Crystal violet (excess crystal violet was removed by clean water rinsing) was dissolved with 0.1 ml of 33% acetic acid, and the absorbance value was detected at 570 nm by a microplate reader.

### 2.9. Transwell

Matrigel was taken out from −20°C in advance and then was placed in the refrigerator at 4°C overnight and melted from the solid state to the liquid state. After being diluted to 1 : 8, the Matrigel was coated on the upper chamber surface of the bottom membrane of the transwell chamber. Then, the transfected cells were digested with 0.25% trypsin, and the cell density was adjusted to 2 × 10^5^/mL. Subsequently, 200 *μ*L of cells was seeded into the upper layer of the transwell chamber to perform serum-free culture. Then, 800 *μ*L of medium containing 10% FBS was added to the wells in the lower layer of the chamber. The cells were incubated in a incubator at 37°C for 24 h to pass through the filter membrane of the chambers. Furthermore, chambers were extracted, and the cells were fixed with 4% paraformaldehyde for 1 h and washed once with PBS. Subsequently, the cells were stained with 0.1% crystal violet for 1 h, washed with distilled water, observed with an upright microscope, and photographed after completely dried.

### 2.10. Statistical Analysis

The obtained experimental data were statistically analyzed using SPSS 24.0 software. The data were expressed with the form of mean ± standard deviation (Mean ± SD). *T*-test or one-way ANOVA was applied for comparisons between two groups or multiple groups. *P* < 0.05 indicated a significant difference. All data were plotted using GraphPad Prism 8.0 software.

## 3. Results

### 3.1. Up-Regulation of FUT7 in Pediatric Patients with Acute Lymphoblastic Leukemia

First, qRT-PCR and western blotting were utilized to determine the FUT7 expression in children with ALL. The results showed that the level of FUT7 mRNA and protein was notably up-regulated in bone marrow samples from children with ALL (Figures 1(a), 1(b)). This result suggested that Fut7 may be involved in the occurrence and development of ALL in children.

### 3.2. Knockdown of FUT7 Significantly Inhibits the Malignant Progression of Acute Lymphoblastic Leukemia Cells

The effect of FUT7 on the malignant progression of ALL cells was further investigated. The results demonstrated a corresponding decrease or increase in FUT7 expression in cells after knockdown or overexpression of FUT7 (Figure 2(a)), indicating good efficiency for cell knockdown or overexpression and availability for the subsequent experiments. Further MTT assay, fibronectin adhesion assay, transwell and flow cytometry results revealed that the cell proliferation rate, adhesion ability and invasion ability were significantly inhibited, and apoptosis was significantly promoted after knockdown of FUT7. However, after overexpression of FUT7, the cell proliferation rate and invasion ability were notably promoted, and apoptosis was significantly inhibited (Figures 2(b)–2(g)). The above results indicated that knockdown of Fut7 inhibited proliferation, adhesion and invasion of Jurkat cells and promoted apoptosis.

### 3.3. Knockdown of Fut7 Significantly Inhibits the Activation of the Integrin/FAK/AKT Pathway in Jurkat Cells

The mechanism of FUT7 affecting the occurrence and development of ALL was further studied. The results revealed that knockdown of FUT7 significantly reduced the protein expression level of integrin *α*5, integrin *β*1, p-FAK and p-AKT pathway-related proteins. However, after overexpression of FUT7, the protein expression level of integrin *α*5, integrin *β*1, p-FAK, and p-AKT in the cells was notably increased (Figures 3(a), 3(b)). The above results indicated that knockdown of Fut7 significantly inhibited the activation of the integrin/FAK/AKT pathway in Jurkat cells.

## 4. Discussion

Acute leukemia (AL) is a malignant clonal disease of hematopoietic stem cells, and the affected cells arrest at an early stage of differentiation and development due to enhanced self-renewal, uncontrolled proliferation, impaired differentiation, and blocked apoptosis. ALL is a very common subtype in AL. In recent years, with the advancement of medical treatment and the emergence of some new treatments, the 5-year disease-free survival rate of ALL has approached 80% [23]. However, about 20% of children still fail to achieve complete remission (CR) or experience relapse after remission.

Tumors are characterized by abnormal cell growth, invasion or spread to other tissues of the body. Abnormal glycosylation of tumor cells is considered to be a common feature of tumor pathogenesis, which often shows abnormal glycoproteins or differential expression of different carbohydrate epitopes [24]. Increased fucosylation and sialylation as well as aberrant O-glycans are recognized characteristics of malignant cell transformation [25]. Overexpression of fucosylated epitopes [e.g., type I (H1, Le^*a*^, Le^*b*^, and *s* Le^*a*^) and type II (H2, Le^*x*^, Le^*y*^, and sLe^*X*^)] frequently occurs on the surface of tumor cells, which is mainly caused by up-regulation of the related FucT expression [24]. The above changes have a great impact on tumors (cell-cell adhesion, cell-matrix interaction, cell signal transduction, metabolism, angiogenesis, and immune regulation), ultimately leading to cancer progression and metastasis. In bladder cancer, down-regulation of FUT7 inhibits the proliferation, migration, invasion, and EMT of bladder cancer cells, while up-regulation of FUT7 shows the opposite effect [20]. In non-small cell lung cancer, FUT7 promotes the proliferation and invasion of A549 cells by activating the EGFR/AKT/mTOR signaling pathway, which is expected to be a potential therapeutic target for non-small cell lung cancer [26]. In this study, FUT7 was found to be highly expressed in ALL patients and could promote the proliferation, adhesion and invasion of Jurkat cells and inhibit cell apoptosis, which was consistent with the results of previous studies.

Integrins, a member of the transmembrane receptor family, are heterodimeric complexes composed of *α* and *β* subunits [27]. The 18 *α* subunits and 8 *β* subunits found now can comprise 24 different integrin protein receptors. The extracellular functional region of integrins is a spherical structure about 20 nm in length. Specifically, the external functional structure mainly binds to extracellular matrix functional proteins, and the internal structure of cells binds to actin. Moreover, both extracellular and internal structures play a role in specific signal transduction pathways and cell-cell adhesion as well as adhesion between cells and epithelial-mesenchymal transition (EMT) [28]. Integrin *α*5 (ITGA5) normally binds to integrin *β*1 (ITGB1) to form integrin *α*5*β*1, which acts as a receptor for cell differentiation, growth and migration. Studies have confirmed that ITGA5 is overexpressed in a variety of human tumors [29, 30], but studies on ITGA5 in ALL were few involved. FUT4 has been found to activate a series of signal transduction mediated by integrin *α*5*β*1 and accelerate adhesion and invasion between integrin *α*5*β*1 and extracellular matrix fibronectin in leukemia cells by increasing glycosylation [31]. In colorectal cancer, hypoxic culture can markedly induce FUT7 and ITGA5 expression in cancer cells [32]. In this study, we also found that overexpression of FUT7 promoted the integrin *α*5 and integrin *β*1 expression in ALL, which is consistent with the results of previous studies.

Focal adhesion kinase (FAK) is a non-receptor tyrosine kinase involved in many important cell biological processes, such as cell adhesion, motility, invasion and metastasis [33]. Besides, FAK is a key upstream protein of cancer-promoting signals such as PI3K/AKT, ERK and MAPK and plays an important role in the invasion and metastasis of various tumors [34]. The above result is consistent with the result in this study that knockdown of FUT7 in ALL cells significantly inhibited the p-FAK and p-AKT expression.

## 5. Conclusion

In summary, this study discovers that FUT7 promotes the adhesion and invasion of ALL cells by activating the integrin/FAK/AKT signaling pathway, resulting in the occurrence and development of ALL. Therefore, the FUT7/integrin/FAK/AKT axis is expected to be a new target for clinical treatment of ALL.

## Figures and Tables

**Figure 1:** FUT7 expression in pediatric patients with acute lymphoblastic leukemia: (a) qRT-PCR was utilized to detect the level of the FUT7 mRNA expression in bone marrow samples in each group (ALL group, *n* = 30; control group, *n* = 10) and (b) western blotting was applied for checking the protein expression level of FUT7 in bone marrow samples from patients in each group,  ^*∗*^ ^*∗*^*P* < 0.01 vs. control group.

**Figure 2:** Effect of knockdown or overexpression of FUT7 on the malignant process of acute lymphoblastic leukemia cells: (a) qRT-PCR was utilized for the test of FUT7 expression in Jurkat cells after knockdown or overexpression of FUT7; (b) MTT assay was performed to detect the cell proliferation ability of Jurkat cells after knockdown or overexpression of FUT7; (c) fibronectin adhesion assay was adopted to check the cell adhesion ability of Jurkat cells after knockdown or overexpression of FUT7; (d) transwell was applied to detect the cell invasion ability of Jurkat cells after knockdown of FUT7; (e) transwell was utilized to detect the cell invasion ability of Jurkat cells after overexpression of FUT7; (f) flow cytometry was used for the detection of the apoptosis of Jurkat cells after knockdown of FUT7; and (g) flow cytometry was used to check the apoptosis of Jurkat cells after overexpression of FUT7.  ^*∗*^ ^*∗*^*P* < 0.01 vs. ShNC or NC.

**Figure 3:** Effect of knockdown or overexpression of Fut7 on integrin/FAK/AKT pathway in Jurkat cells: (a) western blotting was applied for the detection of the expression level of proteins related to the integrin/FAK/AKT pathway in cells after knockdown of Fut7 and (b) western blotting for the determination of the expression level of proteins related to the integrin/FAK/AKT pathway in cells after overexpression of Fut7.  ^*∗*^ ^*∗*^*P* < 0.01 vs. ShNC or NC.

**Table 1:** Primer sequences.

Primer		Sequences (5′-3′)
FUT7	Forward	GAATGAGAGCCGATACCAACGC
	Reverse	TAGCGGTCACAGATGGCACAGA
GAPDH	Forward	GGAGCGAGATCCCTCCAAAAT
	Reverse	GGCTGTTGTCATACTTCTCATGG

## Data Availability

The data used to support the findings of this study are available from the corresponding author upon request.
